The article "Characteristics of Pulse Parameters in Patients with Polycystic Ovary Syndrome Varied at Different Body Mass Index Levels" was published in 2022. Journal: Evid Based Complement Alternat Med.

# Characteristics of Pulse Parameters in Patients with Polycystic Ovary Syndrome Varied at Different Body Mass Index Levels

**DOI:** 10.1155/2022/7220011

**Published:** 2022-05-02

**Authors:** Xiao Feng, Lu Feng, Hui Gao, Qing-Sheng Wang, Yu-Mo Xia, Zhao-Xia Xu, Yi-Qin Wang

**Affiliations:** Basic Medical College, Shanghai University of Traditional Chinese Medicine, Shanghai, China

## Abstract

**Objective:**

To analyze the characteristics of pulse graph parameters in patients with polycystic ovary syndrome (PCOS) varied at different body mass index (BMI) levels and to provide pulse diagnosis basis for syndrome differentiation and treatment of PCOS.

**Methods:**

Pulse graph parameters of 152 patients with PCOS (26 lean patients, 63 patients with moderate weight, and 63 overweight patients) were measured by a Z-BOX pulse meter, and the pulse graph parameters of patients with PCOS varied at different BMI levels were analyzed.

**Results:**

Fine pulse, slippery pulse, and string-like pulse were the most common pulse conditions in patients with PCOS. The common pulse conditions of patients with PCOS varied at different BMI levels. The order of pulse conditions was as follows: lean group: fine pulse > string-like pulse > slippery pulse; moderate group: fine pulse > slippery pulse > string-like pulse; and overweight group: slippery pulse > fine pulse > sunken pulse. Compared to the overweight group, the pulse graph parameters *h*1, *h*3, *h*4, *h*5, *h*4/*h*1, As, and Ad increased in the moderate group (*P* < 0.05), and the parameters *h*1, *h*3, and Ad increased (*P* < 0.05) and the parameter t1 decreased (*P* < 0.05) in the lean group.

**Conclusion:**

Pulse graph parameters among patients with PCOS varied at different BMI levels, which can probably provide pulse diagnosis basis for syndrome differentiation and treatment of PCOS by traditional Chinese medicine (TCM).

## 1. Introduction 

Polycystic ovary syndrome (PCOS) is a common gynecological endocrine disorder, and it is common in females with long-term anovulation, hyperandrogenemia, rare menstruation or even amenorrhea or irregular uterine bleeding, infertility, hirsutism, acne, and other clinical symptoms. Obesity and insulin resistance are also common in patients with PCOS.

Studies have shown that more than 60% of patients with PCOS are overweight or obese [1]. High body mass index (BMI) is not only a risk factor for the occurrence and development of PCOS, but it is also an influencing factor for insulin resistance, spontaneous abortion, pregnancy-related hypertension, low ovarian response, and reduced rate of frozen-thawed embryo implantation in patients with PCOS [2–7]. The relationship between PCOS and BMI has mostly been reported in clinical studies on the association of PCOS with physical and chemical indices, risk factors, clinical phenotypes, and ethnic gene polymorphisms [8–10].

The article "Characteristics of Pulse Parameters in Patients with Polycystic Ovary Syndrome Varied at Different Body Mass Index Levels" was published in 2022. Journal: Evid Based Complement Alternat Med.

With the development and application of pulse diagnosis in objective clinical assessments, the discussion on the characteristics of pulse graph for PCOS is gradually gaining interest among researchers. According to “Pulse Confirmation (mai que, 《脉确》),” obese people are considered to have a deeply located pulse, while thin people have a superficially located pulse, indicating that obesity and leanness affect the pulse of the human body. In the present study, the Z-BOX pulse meter jointly developed by Shanghai University of Traditional Chinese Medicine (SHUTCM) and Shanghai Asia and Pacific Computer Information System Co., Ltd. was used to obtain pulse graph, and the parameters in the time-domain of pulse graph of patients with PCOS varied at different BMI levels were analyzed to provide an objective basis of pulse diagnosis for clinical syndrome differentiation and treatment of PCOS. A study flowchart is shown in Figure 1.

## 2. Methods

### 2.1. Participants

#### 2.1.1. General Condition of Patients

The study included 152 patients with PCOS who were admitted to SHUTCM and Shuguang Hospital affiliated to SHUTCM from August 2018 to March 2021. According to the guidelines for prevention and control of overweight and obesity in Chinese adults, the patients with PCOS were divided into the lean group (BMI <18.5 kg/m^2^, 26 patients), moderate group (18.5 ≤ BMI <24 kg/m^2^, 63 patients), and overweight group (BMI ≥ 24 kg/m^2^, 63 patients) [11]. The blood pressure of these patients was normal.

#### 2.1.2. Inclusion Criteria

Inclusion criteria for patients with PCOS were as follows: (1) patients were diagnosed to have PCOS according to the Chinese guidelines for diagnosis and treatment of polycystic ovary syndrome (2018) [12], where other diseases that may cause hyperandrogenism and abnormal ovulation were excluded, and the patients presented with sparse menstruation, amenorrhea, or irregular uterine bleeding and one of the following two findings: clinical and/or biochemical hyperandrogenism (HA) or polycystic ovarian morphology (PCOM); (2) the age of the included patients ranged between 18 and 40 years; (3) patients had no other apparent gynecological diseases and organic diseases such as liver or kidney disorder; and (4) patient provided informed consent to participate in this clinical study.

#### 2.1.3. Exclusion Criteria

Exclusion criteria were also based on the Chinese guidelines for diagnosis and treatment of polycystic ovary syndrome (2018) [12]. Patients were excluded from the study if they presented any of the following conditions: patients with adenomyosis, Cushing's syndrome, chromosomal abnormalities, congenital adrenal cortical hyperplasia, and chocolate cyst of the ovary; patients with organic lesions of other organs; patients with significant incomplete clinical data; and patients who refused to cooperate.

The article "Characteristics of Pulse Parameters in Patients with Polycystic Ovary Syndrome Varied at Different Body Mass Index Levels" was published in 2022. Journal: Evid Based Complement Alternat Med.

### 2.2. Pulse Collection

The pulse graph information was collected from the guan pulse of the patient's left hand because it pulsates clearly and can be easily detected. The Z-BOX pulse meter was used to collect the pulse graph information of patients with PCOS from 9 AM to 11 AM or from 1 PM to 4 : 30 PM. The patients remained relatively calm and were prohibited to eat, drink, or have violent emotional fluctuations 30 min before the test. The patients assumed the sitting position, and the forearm was naturally spread forward and placed at the same level as the heart. The wrist was kept straight, the palm was maintained upward, the fingers were slightly bent, and a soft pulse pillow was placed under the wrist joint. A series of pulse graphs of three pressure sections within the pulse pressure range of 25–250 g were recorded continuously. The pulse graph for each pressure section was collected for 10 s and recorded continuously for 60 s. The pulse graph with the highest main amplitude, apparent fluctuation of three peaks, and a steep ascending branch without incisure was selected for time-domain parameter analysis. The physiological significance of the pulse graph parameters was determined by referring to “Pulse Diagnosis of Modern Traditional Chinese Medicine” [13].

The pulse graph parameters are shown in Figure 2. Each parameter of pulse graph has its corresponding physiological significance. Parameters *h*1–*h*5 are amplitude parameters and mainly represent the amplitude height. Parameter *h*1 is the main wave amplitude, *h*3 is the tidal wave amplitude, *h*4 is the dicrotic notch amplitude, and *h*5 is the dicrotic wave amplitude. Parameters *t*–*t*5 are the time value parameters and *t* represents a complete pulse cycle. On the sphygmogram, *t*1 is the time value from the start point to the crest point of the main wave, *t*4 is the time value from the start point to the dicrotic notch, and *t*5 is the time value from the dicrotic notch to the end point. Parameter *w* is the width at 1/3 of the main wave. As and Ad are the area parameters: As represents the systolic area and Ad represents the diastolic area. The *h*3/*h*1, *h*4/*h*1, *h*5/*h*1, and *w*/*t* are the ratio parameters. Parameter *h*3/*h*1 mainly reflects vascular wall compliance and peripheral resistance, *h*4/*h*1 reflects the level of peripheral resistance, *h*5/*h*1 mainly reflects aortic compliance and aortic valve function, and *w*/*t* corresponds to the duration of elevated aortic pressure and is related to peripheral resistance.

The article "Characteristics of Pulse Parameters in Patients with Polycystic Ovary Syndrome Varied at Different Body Mass Index Levels" was published in 2022. Journal: Evid Based Complement Alternat Med.

### 2.3. Statistical Analysis

Statistical analysis was performed using IBM SPSS version 25.0. One-way analysis of variance (ANOVA) was used to compare the measurement data that conformed to normal distribution or had an equal variance between groups, while the Bonferroni correction was used for multiple comparison between groups. An independent sample Wilcoxon rank sum test was used to compare the measurement data that did not conform to normal distribution or had an unequal variance. The chi-square test was used to analyze count data between groups. The level of significance was set at *P* < 0.05 for all the analyses.

## 3. Results

### 3.1. Age

The age of patients with PCOS is given in Table 1 and Figure 3. The average age of the patients from the lean, moderate, and overweight groups was 25.423 ± 4.12, 27.603 ± 4.563, and 27.635 ± 4.787 years, respectively. One-way ANOVA showed no significant difference in age among the three groups (*P* > 0.05).

### 3.2. Distribution of Pulse Conditions of Patients with PCOS in the Lean, Moderate, and Overweight Groups

Figure 4 and Table 2 show the pulse conditions of patients with PCOS in the lean, moderate, and overweight groups. Among the 152 patients with PCOS, fine pulse (74.34%) accounted for the highest proportion of pulse condition, followed by slippery pulse (55.92%) and string-like pulse (37.50%). The first three most common pulse conditions were not identical in the different groups of patients with PCOS. According to the order of frequency from high to low, the following trend was noted: lean group: fine pulse > string-like pulse > slippery pulse; moderate group: fine pulse > slippery pulse > string-like pulse; overweight group: slippery pulse > fine pulse > sunken pulse.

### 3.3. Comparison of the Time-Domain Parameters of Pulse Graph among the Lean, Moderate, and Overweight Groups

Tables 3 and 4 provide comparisons of the time-domain parameters of pulse graph among the lean, moderate, and overweight groups. The pulse graph parameters *t*4, *t*5, *t*, *w*, *h*4/*h*1, and *w*/*t* conformed to normal distribution and had an equal variance, and these parameters were analyzed by one-way ANOVA and Bonferroni correction. The pulse graph parameters *h*1, *h*3, *h*4, *h*5, *t*1, As, Ad, *h*3/*h*1, and *h*5/*h*1 did not conform to normal distribution or had an unequal variance, and these parameters were analyzed by the Wilcoxon rank sum test. The results showed that compared to the overweight group, the moderate group showed a significant increase (*P* < 0.05) in the pulse graph parameters *h*1, *h*3, *h*4, *h*5, *h*4/*h*1, As, and Ad, while the lean group showed a significant increase (*P* < 0.05) in the parameters *h*1, *h*3, and Ad and a significant decrease (*P* < 0.05) in the parameter *t*1. No significant differences were observed in the residual pulse graph parameters between the groups (*P* > 0.05).

The article "Characteristics of Pulse Parameters in Patients with Polycystic Ovary Syndrome Varied at Different Body Mass Index Levels" was published in 2022. Journal: Evid Based Complement Alternat Med.

## 4. Discussion

Obesity is not only the clinical manifestation of patients with PCOS but also the influencing factor of the PCOS disease process. An increase in BMI can directly or indirectly have a negative influence on the endocrine level, pregnancy complications, and outcomes of assisted reproduction in patients with PCOS [14–17]. A correlation has been found between female BMI and pulse graph parameters [18]. However, to date, no clinical studies have analyzed the characteristics of pulse graph parameters in patients with PCOS varied at different BMI levels.

The results of the present study showed that fine pulse, slippery pulse, and string-like pulse were the most common pulse conditions in patients with PCOS. Fine pulse is mostly related to the deficiency of qi and blood that leads to inadequate filling and inflation of the artery. The formation mechanism of string-like pulse is related to stressful pulse and pulse path, which is caused by liver dysfunction of dredging and deficiency of qi or blood [19]. According to TCM, liver dysfunction is common in women with constant depressive mood and deficiency of qi and blood. The cause and mechanism of PCOS are related to the dysfunction of the kidney, liver, and spleen. Kidney heavenly tenth or blood deficiency, depressed liver qi running transversely impairs the spleen function in transportation and transformation, and formation of phlegm-dampness can lead to the development of fine pulse, slippery pulse, and string-like pulse.

This study revealed that the pulse conditions of patients with PCOS varied at different BMI levels. At the same BMI level, the top three pulse conditions were not exactly the same. According to the order of frequency from high to low, the lean group showed fine pulse, string-like pulse, and slippery pulse; the moderate group showed fine pulse, slippery pulse, and string-like pulse; and the overweight group showed slippery pulse, fine pulse, and sunken pulse. The distribution of the same pulse condition in patients with PCOS varied at different BMI levels was also different. According to the proportion of pulse conditions from high to low in different groups, the following trend was observed: string-like pulse: moderate group > lean group > overweight group; fine pulse: moderate group > overweight group > lean group; sunken pulse: overweight group > moderate group > lean group.

The article "Characteristics of Pulse Parameters in Patients with Polycystic Ovary Syndrome Varied at Different Body Mass Index Levels" was published in 2022. Journal: Evid Based Complement Alternat Med.

According to TCM, obese people have more phlegm-dampness and deeply located pulse. Slippery pulse and sunken pulse were more common in the overweight group of patients with PCOS and were related to obesity and phlegm-dampness, while string-like pulse was more common in the lean group and was related to stagnation of qi in the liver resulting from impairment of free coursing. However, patients with the proportion of string-like pulse were more likely to have a moderate BMI than a low BMI. It was speculated that this is related to physiological variation. A study found that the formation of physiological string-like pulse was related to the increase in BMI [20]. In the present study, the distribution of fine pulse was not negatively correlated with the BMI level, which may be related to the severity of phlegm-dampness and deficiency of qi and blood in patients with PCOS.

The present study showed that the pulse graph parameters of patients with PCOS varied at different BMI levels. Compared to the overweight group, the moderate group showed a significant increase in the pulse graph parameters *h*1, *h*3, *h*4, *h*5, *h*4/*h*1, As, and Ad, while the lean group showed a significant increase in the parameters *h*1, *h*3, and Ad and a significant decrease in the parameter *t*1. These findings suggested that the left ventricular pumping function and arterial compliance in obese patients with PCOS were worse than those in nonobese patients, and the peripheral resistance of obese patients was also lower than that of nonobese patients; this may be related to the decline in myocardial contractility and cardiac function compensation in obese patients. Previous studies have shown an independent negative correlation between BMI and myocardial contractility [21], and a decrease in myocardial contractility led to a decrease in left ventricular ejection function. Because obesity can lead to cardiac hypertrophy, the heart plays a compensatory role by increasing physiological circulating blood volume and reducing systemic vascular resistance [22].

Recent studies have revealed a chronic inflammatory state in patients with PCOS. BMI and expression levels of serum inflammatory markers, namely, hypersensitive C-reactive protein, procalcitonin, and interleukin-6, were found to be significantly positively correlated, and obesity may increase the correlation between PCOS and inflammation [23, 24]. The decrease in arterial compliance in obese patients with PCOS may be related to arteriosclerosis caused by chronic inflammation.

In conclusion, the results of this study showed differences in the distribution of pulse conditions and pulse graph time-domain parameters in patients with PCOS varied at different BMI levels. These differences were related to stagnation of qi in the liver resulting from impairment of free coursing, degree of phlegm-dampness, deficiency of qi and blood, myocardial dysfunction, and aggravation of chronic inflammation caused by obesity. The present study had three limitations. First, the differences in pulse conditions between patients with PCOS and normal women under the same BMI level were not compared. Second, the age range of the patients was relatively narrow, and the changes in pulse conditions at different age stages were not analyzed. Third, the sample size was small, and patient distribution among groups with different BMI levels was uneven. In the follow-up study, we will increase the sample size for in-depth research in order to provide an objective basis for the use of pulse graph to guide syndrome differentiation and treatment of PCOS by TCM.

The article "Characteristics of Pulse Parameters in Patients with Polycystic Ovary Syndrome Varied at Different Body Mass Index Levels" was published in 2022. Journal: Evid Based Complement Alternat Med.

## Figures and Tables

**Figure 1:** Study flowchart.

**Figure 2:** The amplitude, time, and area of the pulse graph.

**Figure 3:** Box plot of age distribution of 152 patients with PCOS.

**Figure 4:** The distribution of pulse condition in 152 patients with PCOS.

**Table 1:** The age of patients with PCOS (*n* = 152).

Variables	Lean group (*n* = 26)	Moderate group (*n* = 63)	Overweight group (*n* = 63)	*P* value
Average age	25.423 ± 4.12	27.603 ± 4.563	27.635 ± 4.787	0.088
Minimum age	18	19	18	-
Maximum age	32	39	40	-

The data are represented as the mean ± standard deviations.

**Table 2:** Frequencies of patients with PCOS in lean, moderate, and overweight groups (*n* = 152).

Variables	Lean group (*n* = 26)	Moderate group (*n* = 63)	Overweight group (*n* = 63)
Floating pulse	0 (0.00)	0 (0.00)	1 (1.59)
Sunken pulse	0 (0.00)	3 (4.76)	25 (39.68)
String-like pulse	17 (65.38)	27 (42.86)	13 (20.63)
Slippery pulse	10 (38.46)	30 (47.62)	45 (71.43)
Fine pulse	22 (84.62)	56 (88.89)	35 (55.56)
Rapid pulse	3 (11.54)	7 (11.11)	12 (19.05)
Weak pulse	0 (0.00)	5 (7.93)	0 (0.00)

The data are represented as the frequency (percentage).

**Table 3:** Comparison of pulse graph parameters among lean, moderate, and overweight groups (*n* = 152).

Variables	Lean group (*n* = 26)	Moderate group (*n* = 63)	Overweight group (*n* = 63)	*P* value
*t*4	0.072 ± 0.022	0.076 ± 0.020	0.073 ± 0.022	0.520
*t*5	0.151 ± 0.027	0.150 ± 0.036	0.145 ± 0.035	0.637
*w*	0.061 ± 0.014	0.061 ± 0.016	0.060 ± 0.015	0.861
*t*	0.219 ± 0.022	0.226 ± 0.035	0.217 ± 0.032	0.276
*h*4/*h*1	0.299 ± 0.142	0.332 ± 0.139^Δ^	0.265 ± 0.150	0.036
*w*/*t*	0.280 ± 0.054	0.270 ± 0.051	0.274 ± 0.049	0.651

The data are represented as the mean ± standard deviations. Compared with the overweight group, ^Δ^*P* < 0.05.

The article "Characteristics of Pulse Parameters in Patients with Polycystic Ovary Syndrome Varied at Different Body Mass Index Levels" was published in 2022. Journal: Evid Based Complement Alternat Med.

**Table 4:** Comparison of pulse graph parameters among lean, moderate, and overweight groups (*n* = 152).

Variables	Lean group (*n* = 26)	Moderate group (*n* = 63)	Overweight group (*n* = 63)	*P* value
*h*1	55.926 (37.068, 66.888)^Δ^	56.888 (37.202, 65.226)^ΔΔ^	40.254 (25.843, 50.723)	<0.01
*h*3	42.753 (32.424, 56.366)^ΔΔ^	43.126 (29.512, 52.820)^ΔΔ^	30.698 (20.296, 42.191)	<0.01
*h*4	14.412 (8.861, 25.130)	16.843 (11.115, 25.017)^ΔΔ^	8.961 (4.894, 17.058)	<0.01
*h*5	21.105 (10.346, 31.799)	25.909 (18.258, 32.548)^Δ^	18.589 (11.460, 28.332)	0.020
*t*1	0.041 (0.039, 0.044)^Δ^	0.043 (0.041, 0.046)	0.045 (0.041, 0.049)	0.110
As	1366.125 (921.447, 2114.489)	1736.219 (956.143, 2200.505)^ΔΔ^	978.471 (558.252, 1746.957)	0.002
Ad	2097.540 (1335.111, 2787.269)^ΔΔ^	2043.218 (1358.543, 2604.711)^ΔΔ^	1346.452 (800.123, 2096.211)	0.001
*h*3/*h*1	0.848 (0.737, 0.901)	0.826 (0.751, 0.869)	0.823 (0.742, 0.862)	0.451
*h*5/*h*1	0.439 (0.247, 0.545)	0.479 (0.407, 0.550)	0.493 (0.370, 0.624)	0.313

The data are represented as the median (quartile). Compared with the overweight group, ^Δ^*P* < 0.05, ^ΔΔ^*P* < 0.01.

## Data Availability

The Ethics Committee of Shanghai University of Traditional Chinese Medicine limited the measurement data used to support the results of this study in order to protect the privacy of patients. For researchers who meet the criteria for obtaining confidential data, the data of this study are available from the corresponding author upon request.
